# Applying Lightweight Deep Learning-Based Virtual Vision Sensing Technology to Realize and Develop New Media Interactive Art Installation

This article has been retracted.

**DOI:** 10.1155/2022/9119316

**Published:** 2022-07-11

**Authors:** Lanjun Luo

**Affiliations:** Cutting Edge Imaging College, Chung-Ang University, Seoul 156756, Republic of Korea

## Abstract

The work intends to optimize the situation that interactive art devices and remote control based on traditional technology cannot meet people's actual needs to a certain extent. With the assistance of Lightweight Deep Learning (LDL) models, Interactive Artistic Installation (IAI) shows excellent creative potential in terms of dimension, space, and sense. Virtual Vision Sensing Technology (VST) explores the emotional semantics in the human-machine environment with the help of interactive art, finds the emotional interaction elements between human and machine, and promotes Human-Computer Interaction (HCI). From the perspective of the media elements of interactive art, this paper reviews the virtual VST that subverts the expression of interactive art. Then, from the perspective of artistic creation, the impact of virtual VST on IAI thinking, methods, and artistic experience is analyzed. Thereupon, a scene construction method is designed where the physical equipment is premodeled. The model is loaded in real time with visual information. The proposed method does not require complex vision and laser scanning equipment or high-configured computer systems. The proposed new media IAI model realizes the real-time loading of the scene model. According to the physical equipment dynamic information obtained by the visual data acquisition system, the proposed method can keep the virtual scene and physical models in motion synchronization. Finally, experiment results corroborate that the environment will significantly interfere with the experimental results. The training data set with boundary occlusion will be more suitable for model training and better test results (about 97% accuracy). Hence, the research content can make the Virtual Reality works have better performance, especially the sense of experience from the perspective of aesthetics. Meanwhile, it also enriches the research theory in the field of new media art installation technology.

## 1. Introduction

Unlike other art forms, interactive art's uniqueness lies in the “situation” constructed by the artistic works. In simpler terms, interactive artists engage viewers as part of the work and who help complete the work [1]. The concept of interaction between works of art and viewers is an age-old problem. Researchers' interest in interactive art has not been rekindled until the Deep Learning (DL) technology boomed in the twenty-first century. Since then, artists' aspiration has been sublimed from spiritual-level viewer-art interaction to the viewers' participation and immersion in the art design [2–4]. Technologically speaking, interaction is omnipresent in real life. It has also had a particular impact on the advancement of science and the betterment of human well-being. For example, many Social Media Platforms (SMPs) like Taobao, Alipay, and WeChat have fundamentally changed people's habits and lifestyles. In particular, Virtual Reality (VR)-based Interactive Art Installation (IAI) involves multiple disciplines. From the perspective of creators and designers, IAI can structure artistic works, improve User Experience (UX), and consummate the quality of artistic works [5, 6].

Globally, virtual Vision Sensing Technology (VST) and IAI originated in the 1960s. A series of new artistic concepts have been formulated, such as “natural intelligence,” “cyber art,” “and “artificial life art.” Zhou (2020) pointed out that, under the information age, new media interactive art was rising rapidly. New media interactive art combines art design with other technologies. New media interactive art can not only repair and reproduce damaged traditional cultural resources, but also use virtual VST to show cultural venues and protect and disseminate precious cultural resources. Compared with the protection and dissemination of other traditional cultural resources, new media interactive art has a protective effect on other traditional cultural resources in different forms. By giving full play to the application advantages of new media interactive art, it provides important technical support for historical and cultural researchers. Audio visualization is an objective interpretation and judgment of music performance. It is a way of understanding, analysing, and comparing music performance ability and internal structure. As a way of expression of new media art, audio visualization has been widely used and appreciated from large-scale lighting performance, stage performance to music video [7]. Johnson et al. (2019) took cyberspace as an example to illustrate the planning, design, and production of audio visualization in new media art products. In addition to the creative source, product naming, style definition, music selection and editing, scene design, and interaction design, they also briefly introduced the software and hardware resources used in product creation [8]. Joshi et al. (2021) established a complete theoretical system of machine vision, which divided visual processing into two-dimensional data acquisition, key element extraction, and three-dimensional reconstruction. According to the point, line, curvature, and other elements of the image and the relationship between various elements, the three-dimensional information of the scene was restored through a series of postprocessing [9]. From different perspectives, experts and scholars put forward their own views on the implementation and development of virtual VST in the new media IAI technology, which provides rich theoretical results for the future research in this field. However, the deficiency is that it only cuts in from a single perspective and has not comprehensively analyzed the impact of VST on IAI.

Traditional art creation mainly relies on daily experience, intuitive judgment, and visual observation. However, with the development of Artificial Intelligent (AI) technology and changes in audience aesthetics, artists need to have a new understanding of artistic creation and receive new creation techniques, concepts, and terminology. Based on previous research, this paper analyzes the technologies involved in new media IAI, such as VR technology and intelligent robot technology. It develops a new media IAI system based on virtual VST. Thereby, the finding enriches the new media IAI methods. The innovation is to design a scene construction method of premodeling of physical equipment and real-time loading of the model combined with visual information, which simplifies the recognition algorithm and improves the recognition accuracy. In addition, this work integrates several proposed key technologies. According to the operation state information of the physical equipment obtained by the visual data acquisition system, this method can keep the motion synchronization between the virtual scene model and the physical model, which provides a methodological reference for the follow-up research in this field to a certain extent.

## 2. Virtual VST Based on Lightweight Deep Learning Model

### 2.1. VR Technology

#### 2.1.1. Basic Concepts and Features

VR, also known as “spiritual technology,” refers to constructing a virtual simulation system through computer technology. Users can immerse in the virtual environment and process various complex information through computer processing to realize the information visualization process [10]. VR technology includes four basic features: imaginativeness, interactivity, immersion, and multisensitivity. The specific attribute of each feature is shown in Table 1.

A VR system generally incorporates a display device, a computer processing system, a virtual environment system, and various interactive systems, such as a haptic system, taste, and speech recognition system. The Human-Computer Interaction (HCI) and the virtual environment are implemented by coordinating multiple systems to restore an immersive user experience in the virtual environment [13, 14].  Figure 1 details the VR system structure.

#### 2.1.2. Basic Type

Depending on the form of participation and the number of participants, VR technology can be subdivided into four categories, as shown in Figure 2.

Desktop Virtual Reality (DVR) uses other monitors or computer screens as the carrier to display the virtual world, and the user controls the virtual characters' actions through the physical controller. DVR features a low-cost and straightforward structure and thus is convenient for market promotion. Nevertheless, since user operations are completed in the physical world, the user feels less immersive, and UX is relatively poor [15].

By contrast, the Immersive Virtual Reality (IVR) system delivers a life-sized virtual environment. Users' viewpoint is traced using the sensory tracking system, such as data gloves and head-worn devices. In this way, the virtual surrounding will be convincing enough for users to engage themselves in the digital world. Inevitably, the IVR system features high costs and is thus hard to be popularized.

The Distributed VR system enables multiple users' simultaneous interaction and information sharing through the Internet in the same VR system. In particular, the Augmented Reality (VR) virtual system is the product of combining the natural environment and the virtual environment. It can enhance users' real-world experiences by imposing sound, touch, and even smell in the virtual world.

#### 2.1.3. Application Status

Since its research and development, VR technology has seen broad applications in all walks of life with strong inclusiveness and functionality. VR can be used to train soldiers or develop and test other frontier technologies in a virtual environment. Doing so can avoid possible danger in the real world, thus guaranteeing personnel security while substantially cutting the cost. The main application areas of VR technology are given in Figure 3.

VR technology can be used for product sales and promotion in the commercial field. For example, in the tourism industry, using VR systems, users can experience famous scenic spots in various regions without leaving their homes. In the real estate industry, customers can have a comprehensive view of the house they are interested in and make multidimensional comparisons before making the final decision. This saves time for both buyers and agents [16, 17]. Further, VR is now used to build a human model for doctors to have an in-depth understanding and stereoscopic view of the structural characteristics of the human body. Some surgical training is also being controlled in a virtual environment, thereby cultivating high-quality physicians and reducing surgery risks.

### 2.2. Emotional HCI Technology

HCI considers the relationship between humans and computers to enhance human cognition, control, and perception of the external world and other natural interaction capabilities. In the field of HCI research, human emotional elements, as the basic elements, play a crucial role, and it is the material signal of Affective Computing (AC). Emotional HCI technology is based on the study of human emotion semantics. It tries to enhance the human-like nature of computer language and endow people's kindness, nature, and other emotions to machines [18, 19]. LDL modeling is a vital technological vehicle for computer emotional cognition. Integrating the LDL model and HCI technology has resulted in more natural multimodal emotional interaction technology, voice emotional interaction technology, and facial recognition interactive technology.

Humans mainly perceive objects that exist objectively through vision. LDL-based HCI models train machines with perceptive vision systems so that the machine can perceive the surroundings and give corresponding feedback. Machine Vision (MV) technology has been widely used in many fields, such as body behavior, emotional interaction, and facial expression recognition [20–22]. Behavioral symbols and facial expressions, as human nonverbal expressions, can give away human emotional and psychological content more vividly and straightforwardly than words. The composition of the MV system is illustrated in Figure 4.

American psychologist Melabin believes humans communicate 55% of the information through body movements and facial expressions. In comparison, the auditory system can only transmit about 38%. Free emotions and the intuition and perception of human spiritual civilization are the sources of art, so integrating AC-based MV into IAI can enhance the emotional connection between things [23].

### 2.3. Visual Marker Localization (VML) Algorithm Based on LDL Model

In the past, cameras could only capture a planar image. The three-dimensional (3D) spatial position of the visual mark must be obtained to obtain the position and motion state of the target. Theoretically speaking, it is possible to infer the 3D coordinates of the visual mark using its planar positions in multiple two-dimensional images. This paper designs a VML method based on a multilayer neural network (MLNN). It is quite different from the traditional multi-eye VML method by considering the mapping relationship of multiple planar coordinates to calculate the 3D coordinates [24, 25].

Essentially, mapping a planar image into 3D coordinates is a regression prediction problem, wherein MLNN is most commonly used. An MLNN is a neural network (NN) with an input layer, an output layer, and multiple hidden layers. Each layer contains multiple nodes, and each node constitutes a perceptron. The output is controlled within a certain range while making discrete values continuous.

#### 2.3.1. Training Sample Generation

A supervised NN must prepare sufficient labeled sample data to train an MLNN. The sample data consists of an input variable and an output variable. Input variables are the radius and planar coordinates of visual markers (VMs), and the 3D spatial coordinates of VMs are output scalars. In that, a training sample can be obtained as [(*x*_1_, *y*_1_, **r**_1_, *x*_2_, *y*_2_, **r**_2_ … *x*_*n*_, *y*_*n*_, **r**_*n*_), (*X*, *Y*, *Z*)]. Apparently, the training data has been decremented through VM simplification. The number of training samples mainly depends on the targets' motion cycle and the camera's sampling frequency. Usually, manual operation is used to collect training samples, which is less time-effective given the large-scale data requirement of NN training [26–28]. Against such a dilemma, the proposed VML method employs an automated sample data generation process.

#### 2.3.2. The NN Training

Set 80% of the training samples as the training set and 20% as the test set. The training set is used to train the neural network, and the test set is used to test and evaluate the neural network after training [29]. The training set and test set are represented by the following equations, respectively:

(1) $$\begin{array}{c} \left[\left(x_{1}^{\text{train}},y_{1}^{\text{train}},r_{1}^{\text{train}},x_{2}^{\text{train}},y_{2}^{\text{train}},r_{2}^{\text{train}}\ldots x_{n}^{\text{train}},y_{n}^{\text{train}},r_{n}^{\text{train}}\right),\left(X^{\text{train}},Y^{\text{train}},Z^{\text{train}}\right)\right], \end{array}$$

(2) $$\begin{array}{c} \left[\left(x_{1}^{\text{t}\theta },y_{1}^{\text{test}},r_{1}^{\text{test}},x_{2}^{\text{test}},y_{2}^{\text{test}},r_{2}^{\text{t}est}\ldots x_{n}^{\text{test}},{\text{y}}_{n}^{\text{test}},r_{n}^{\text{test}}\right),\left({\text{X}}^{\text{test}},{\text{Y}}^{\text{test}},{\text{Z}}^{\text{te}}\right)\right]. \end{array}$$

Equations (1) and (2) represent the training set and test set of neural network, respectively, and [(*x*_1_, *y*_1_, *r*_1_, *x*_2_, *y*_2_, *r*_2_ … *x*_*n*_, *y*_*n*_, *r*_*n*_), (*X*, *Y*, *Z*)] is a training sample. The activation function setting is shown in the following equation:

(3) $$\begin{array}{c} h\left(x\right)=\text{max}\left(0,x\right)=\left\{\begin{array}{c} x\left(x\geq 0\right),\\ 0\left(x<0\right). \end{array}\right. \end{array}$$

In equation (3), *h*(*x*) represents the activation function. The input data of the neural network is weighted and summed by each node, and the offset value is added to obtain the following equation:

(4) $$\begin{array}{c} a_{j}=\sum_{i}w_{ji}x_{i}+b_{j}. \end{array}$$

*j* is node *j* in this layer neural network; *i* is node *i* in the previous neural network; **w**_*ji*_ is the connection weight between nodes *j* and *I*; *x*_*i*_, **b**_*j*_ are the *i*th input and offset value of this node. The final output of the node needs to be processed through the activation function. After substituting equation (4) into the activation function, the following equation is obtained:

(5) $$\begin{array}{c} Z_{j}=h\left(\sum_{i}w_{ji}x_{i}+b_{j}\right)m_{j},m_{j}∼\text{Bernoulli}\left(1-P\right). \end{array}$$

**m**_*j*_ is a parameter conforming to Bernoulli probability distribution. When **m**_*j*_=0, the output value of the node is 0, and the node is deleted. The finally output neural network is the three-dimensional coordinates (*X*, *Y*, *Z*) of the visual mark. The specific value is calculated as follows:

(6) $$\begin{array}{c} X=G_{1}\left(W,B,M\right), \end{array}$$

(7) $$\begin{array}{c} Y=G_{2}\left(W,B,M\right), \end{array}$$

(8) $$\begin{array}{c} Z=G_{3}\left(W,B,M\right). \end{array}$$

In equations (6)–(8), *W* is weight *w* vector, *B* is bias *w* vector, and *M* is mask *m* vector. The training process of neural network can be regarded as the process of gradient descent, and the training errors are shown as follows:

(9) $$\begin{array}{c} E_{X}=\frac{1}{n}\sum_{i}{\left(X-X^{\text{train}}\right)}_{i}^{2}, \end{array}$$

(10) $$\begin{array}{c} E_{Y}=\frac{1}{n}\sum_{i}{\left(Y-Y^{\text{train}}\right)}_{i}^{2}, \end{array}$$

(11) $$\begin{array}{c} E_{Z}=\frac{1}{n}\sum_{i}{\left(Z-Z^{\text{train}}\right)}_{i}^{2}. \end{array}$$

**E**_*X*_, **E**_*Y*_, and **E**_*Z*_ represent the training error of *X,Y*, *Z* coordinates, *n* represents the number, and the meaning of the remaining letters is the same as the above equations. Equations (9)–(11) represent the calculation method of training error of three-dimensional coordinates (*X*, *Y*, *Z*): sum the square of the difference between the original coordinates (*X*, *Y*, *Z*) and the training coordinates (*X*, *Y*, *Z*), divide the obtained number by the number of training, and the final result is the corresponding training error.

The gradient calculation of error is shown in the following equations:

(12) $$\begin{array}{c} \nabla_{W_{n}}^{1/n}{\left\|G_{1}\left(W,B,M\right)-X^{\text{train}}\right\|}_{2}^{2}, \end{array}$$

(13) $$\begin{array}{c} \nabla_{B}\frac{1}{n}{\left\|G_{1}\left(W,B,M\right)-X^{\text{train}}\right\|}_{2}^{2}, \end{array}$$

(14) $$\begin{array}{c} \nabla_{W}\frac{1}{n}{\left\|G_{2}\left(W,B,M\right)-Y^{\text{train}}\right\|}_{2}^{2}, \end{array}$$

(15) $$\begin{array}{c} \nabla_{B}\frac{1}{n}{\left\|G_{2}\left(W,B,M\right)-Y^{\text{train}}\right\|}_{2}^{2}, \end{array}$$

(16) $$\begin{array}{c} \nabla_{W}\frac{1}{n}{\left\|G_{3}\left(W,B,M\right)-Z^{\text{train}}\right\|}_{2}^{2}, \end{array}$$

(17) $$\begin{array}{c} \nabla_{B}\frac{1}{n}{\left\|G_{3}\left(W,B,M\right)-Z^{\text{train}}\right\|}_{2}^{2}. \end{array}$$

The gradient of error is the partial derivative of parameters *W*, *B*, where *M* is a preset parameter, and the meaning of the remaining letters is the same as that of the above equations. After the training samples are substituted into the iterative operation, the weight vector *W* and offset value vector *B* are finally determined; that is, the training of the neural network is completed. After the training, the test samples can be substituted to verify the effectiveness of the neural network.

### 2.4. Virtual Vision Sensing Technology

Vision is key to information acquisition: 80% of all information is obtained through visual means. This section proposes a VST-based information acquisition method to provide a real-time data feed service for VR systems and synchronize the motion state of 3D models and physical entities in real time. The vision-based information acquisition has several advantages. (1) It is a noncontact data acquisition method without altering the original equipment. (2) The sampling frequency of the visual equipment is high, which can be well lent to the HCI and Remote Control System (RCS) in the VR environment. (3) The visual equipment is easy to install, inexpensive, and ready-available visual algorithms. The related research is relatively mature. The proposed method can collect the state information of physical entities, such as position, attitude, and motion, as portrayed in Figure 5.

Figure 5 displays that the interactive art design device method first attaches the predesigned visual mark with significant image features to the measured object and arranges multiple cameras to shoot the measured object from different positions and angles. When the object drives the visual mark to move, the camera captures multiple target object images. The recognition algorithm finds the position and size of the visual mark from the image and transmits the data to the target positioning algorithm based on neural network as the input data of the neural network. The trained neural network algorithm will calculate the spatial three-dimensional coordinate position of the visual mark on the target object according to the input data. According to the three-dimensional coordinate position with visual mark, the spatial coordinate position of the moving part is obtained indirectly. Finally, the corresponding virtual model is driven to keep synchronous motion according to the spatial coordinate data of each moving part in the scene.

## 3. Implementation of New Media Interactive Art Design Device Technology under Virtual Vision Sensing Technology

### 3.1. Real-Time Construction of Virtual Scenes

#### 3.1.1. Virtual Scene Construction Approach

The real scene and the virtual model are isolated in the virtual scene. When the real scene changes, the virtual environment must also change accordingly. During this process, the following issues need to be addressed:

One is the problem of model construction. In modeling physical entities, manual operations often waste much time and energy. It is challenging to complete highly dynamic scene modeling only by manual operations, and automated methods must be used in modeling. However, it is not easy to perform global scanning and 3D reconstruction of real scenes.

The second is the synchronization between the virtual model and the real scene. The real scene is a dynamic changing process, which determines the dynamic features of the physical entities in the virtual scene as well.

The third is the scene loading delay, as depicted in Figure 6.

Modeling and loading involve large amounts of data, which becomes especially obvious in a dynamic change process. This results in screen delay that impacts the interactive experience of the virtual environment.

In order to avoid the above problems, premodeling is proposed for the scene, as demonstrated in Figure 7.

Firstly, the physical entities in the real scene are premodeled. Then, the dynamic objects are visually marked, and the spatial positions of the dynamic objects are captured through visual acquisition. Then, the spatial positions and postures of the dynamic objects are determined using virtual VST. Afterward, the premodeled 3D model is loaded into the virtual scene.

#### 3.1.2. Build Model Physics Driver

The scene model built-in Unity3D is static. Thus, the static model must be made adjustable according to the physical entity's positions. In order to do so, a physical driver script is added to the static model. Unity3D provides multiple sets of instructions to control the model's movement and control the model's position in each frame by calling these instructions in the program.

1. The Transform component controls the model movement. The Transform component can control the model's spatial position, angle, scale, and other states. Unity3D gives objects a Position attribute. Through the Transform.Translate instruction of the Transform component, the coordinate of the Position is adjusted, thereby adjusting the object's position in the scene. The Transform.Translate instruction simplifies the coordinate transformation of moving targets. By adjusting the target's spatial position in each frame, the Unity3D realizes the Motion Effects.
2. The Rigidbody component controls the model movement. Rigidbody is a rigid body component in Unity3D, used to control the physical properties of an object, such as gravity, elastic coefficient, and motion after impact. Rigidbody component's Rigidbody.MovePosition, Rigidbody.AddForce, and Rigidbody.velocity instructions can control the object movement. Specifically, the Rigidbody.velocity can give the object a linear speed. An object's spatial position is controlled by adjusting its speed. By comparison, Rigidbody.AddForce can apply a force to the object to move. Lastly, the Rigidbody.MovePosition is similar to Transform.Translate: the object can be controlled to move left and right up and down.
3. The Character Controller component controls the model movement. The Character Controller can control the characters' positions and adjust users' position changes in the virtual scene. Concretely, Character Controller.SimpleMove can control the character's forward and backward jumping, gravity, and other motion states. The Character Controller.Move can process the physical information that the character needs to handle when moving in space, such as collision and force.

### 3.2. 3D Display Technology Implementation

#### 3.2.1. 3D Glasses

Based on the principle of human stereoscopic vision, this section chooses the 3D glasses to separate the left and right eyes to produce parallax, as showcased in Figure 8.

Figure 8 suggests that the structure of new media 3D stereoscopic display glasses includes two convex lenses and the display screen. The main function of the convex lens makes the picture distance of the display screen longer. The human eye has a zoom function, and the focal length range is 10 cm–30 m. Therefore, the image within 10 cm from the human eye cannot be imaged on the retina. The imaging process of convex lens is shown in Figure 9.

#### 3.2.2. Construction of Display System Based on HTC VIVE

HTC VIVE is a VR head-mounted display product jointly developed by HTC and Value. It is also a VR experience platform with the best display effect and robust versatility. Its display system is revealed in Figure 10.

HTC VIVE display system includes two laser locators for spatial positioning, two operating handles, and a helmet mounted display. There are two display screens in the helmet mounted display, which project images to the left and right eyes, respectively. Each display has the resolution up to 1080 × 1200, which can provide projection display with high definition and large viewing angle. The refresh frame rate of HTC VIVE display is up to 90 frames per second. The high frame rate makes the picture load faster. When the user moves with the display helmet, the picture will not get stuck. To make the equipment thinner, the lens of HTC VIVE is two Fresnel lenses. Compared with ordinary convex lens, Fresnel lens retains the surface curvature of convex lens, removes the lens area that does not participate in refraction, and makes the lens lighter and thinner. HTC VIVE uses a lighthouse laser locator. The two space locators emit infrared laser beams like lighthouses. The sensors on the helmet mounted display and the joystick receive the light emitted by the lighthouse and calculate their position in space according to the angle of the light beam. When the user moves in the space, the helmet display system refreshes the display screen according to its own spatial position and provides the current field of view screen to the user.

Unity3D provides good support for the development of virtual VST. Developing HTC VIVE on the Unity3D platform first installs the SteamVR software on the computer. SteamVR provides a VR running environment and realizes the connection between Unity3D and HTC VIVE hardware. Then, it starts the hardware in SteamVR and sets parameters, such as the connection between the lighthouse and the helmet reality device and the size of the room's activity space. After the SteamVR installation is complete, the Steam VR Plugin is imported into Unity3D. Steam VR Plugin is a VR development kit. The Application Programming Interface (API) in the SteamVR Plugin can be called from Unity3D. In Unity3D, all development is directed towards this API.

The scene model in Unity3D is displayed in the HTC VIVE helmet display and produces a relatively stereoscopic and immersive scene. It is necessary to generate two views, which are displayed on the left and right screens of the helmet display and projected to the left and right eyes. The two views will form a parallax similar to the human eye by deploying two cameras in the Unity3D scene. The two cameras correspond to the human's left eye and right eye, and the horizontal distance between the cameras is equal to the interpupillary distance.

The image size is set to 100 × 100, and at the same time, labels are set for the test data to analyze the experimental results. Then, training steps are set to 10,000, and 100 samples will be selected every 100 steps to calculate the accuracy of the test set. Two comparative experiments with and without environmental elements are carried out. Each experiment will be conducted with and without boundary occlusion.  Figure 11 compares the experiment results.

The comparison between Figures 11(a) and 11(b) reveals that the environment will significantly interfere with the analysis of experimental results, and the accuracy of processing without adding occlusion can reach about 90%. Then, from the results after adding boundary occlusion, for the test data set with common boundary occlusion, using the training data set with boundary occlusion is more targeted to achieve better test results, and the accuracy can reach about 97%.

## 4. Discussion

To study the new media IAI technology, based on the relevant theories such as Lightweight Deep Learning model and virtual VST, this work studies the key technologies required for remote control of equipment in VR environment, including vision-based data acquisition technology, scene real-time construction, and 3D reality technology, and draws the corresponding conclusions. The VR system for pilot training developed by Jeon et al. (2021) can immerse the pilot in the virtual cabin environment. The virtual cabin draws the virtual scene in real time according to the pilot's operation, so that the pilot has a Human-Computer Interaction (HCI) environment like the real driving environment, which greatly reduces the pilot's training cost [30]. The Da Vinci surgical robot system jointly developed by Nasimi et al. (2022) uses a variety of HCI and remote control technologies. The system collects human manipulation information and tactile information, which are processed and transmitted to the manipulator to perform surgical action. The imaging system of the manipulator collects and amplifies the visual signal and transmits it to the VR imaging system to present the surgical scene to the operator in three dimensions [31]. Starting from different fields, the two scholars analyzed the application of virtual technology in real life. However, only from the aviation and medical aspects, there is no research on other fields, and there is a lack of certain universal applicability. In this work, the virtual VST is applied to the new media IAI, which not only enriches the theoretical development of the new media industry, but also provides some conclusions and methods. The disadvantage is that the system has not been put into the specific application environment. Therefore, this should also be strengthened in the follow-up research.

## 5. Conclusion

In the process of human history and civilization, the evolution of artistic expression is closely related to the progress of science and technology. From the perspective of interactive art media elements, this work combs the virtual VST that subverts the expression of interactive art. Then, from the perspective of artistic creation, this work analyzes the impact of virtual VST on interactive artistic creation thinking, creative means, and artistic experience. A scene construction method of premodeling physical equipment and real-time loading model is designed combined with visual information. This method does not need complex visual and laser scanning equipment and high configuration computer system, and the accuracy can reach 97%. In addition, the principle of human eye stereo imaging and spectacle stereo display are studied. Using spectacle VR display technology and HTC VIVE display, the real-time scene is projected to the left eye and right eye, respectively, and the immersive stereo display is realized. Therefore, the research on the realization and development of virtual VST based on Lightweight Deep Learning model in new media IAI technology provides some ideas for the development of this field in the future and can promote the development of new media industry to a certain extent.

However, this work only preliminarily establishes the new media IAI system under the VR environment and opens some technical joints necessary for the system. Relevant research and system functions still need to be developed and improved in the future research, for example, the recognition and location technology of visual markers. The recognition and positioning of visual marks of a new media art device are realized. The research and experiment of multiple visual marks carried by multiple devices in the same space need to be improved.

## Figures and Tables

**Figure 1:** VR system.

**Figure 2:** VR classification.

**Figure 3:** Application fields of VR technology.

**Figure 4:** The composition of the MV system.

**Figure 5:** Frame diagram of IAI.

**Figure 6:** Scene loading delay.

**Figure 7:** Scene construction in real time.

**Figure 8:** 3D glass display structure diagram.

**Figure 9:** Imaging process of the convex lens.

**Figure 10:** HTC VIVE display system.

**Figure 11:** Accuracy of training results. (a) Accuracy with environmental elements. (b) Accuracy without environmental elements.

**Table 1:** Basic features of VR technology.

Feature	Attribute
Imaginativeness	Imaginativeness, also known as autonomy, means that the imaginable space of VR technology is very broad, which can broaden the scope of human cognition. Using VR, people can reproduce real-life scenarios and surreal digital environments [11].
Interactivity	It refers to the degree to which users can get feedback from the environment and the operability of the objects in the virtual environment.
Immersiveness	Immersiveness is also known as immersion. VR technology is to build a real environment in a virtual system through a computer and network system. The real scene is the basis on which the virtual environment is generated. In particular, immersion refers to the degree to which the user feels too real to distinguish the virtual world from the real-life scenes. The goal is to enable users to devote themselves to the virtual environment [12] fully.
	Multisensory refers to that VR technology includes visual perception and traditional computer vision and includes tactile perception, motion perception, force perception, and auditory perception. Perfect VR technology expects to generate all-inclusive perception systems in a virtual system. However, only perception systems, such as touch, hearing, vision, and movement, have been ensembled due to technical limitations

## Data Availability

The data used to support the findings of this study are included within the article.
